# Prevalence of Work-Related Health Hazard and Associated Factors among Health Workers in Public Health Institutions of Gambella Town, Western Ethiopia: Cross-Sectional Survey

**DOI:** 10.1155/2022/6224280

**Published:** 2022-08-29

**Authors:** Ewnetu Ayenew, Wakuma Akafu, Dawit Wolde Daka

**Affiliations:** ^1^Gambella Town Health Office, Gambela, Gambella, Ethiopia; ^2^Department of Health Policy and Management, Faculty of Public Health, Institute of Health, Jimma University, Jimma, Oromia, Ethiopia

## Abstract

**Background:**

Many health-related occupational hazards confront healthcare workers. Examining the prevalence of hazards enables to search for better risk management for healthcare workers because these workers are often the first point of interaction, particularly in resource-limited settings like Ethiopia. Therefore, this study assessed the prevalence of work-related occupational hazards and identified related factors among healthcare workers in public health facilities of Gambella town, Western Ethiopia.

**Methods:**

Institution-based cross-sectional study was conducted among 260 randomly selected healthcare workers from June 1-21, 2021. A semi structured tool was used to collect data and data analysis was performed using SPSS version 25. Multivariable logistic regression was used to identify the predictors of outcome variable and the significance of associations was declared by using a 95% CI and a *p*-value of <0.05.

**Results:**

The prevalence of occupational health hazards among healthcare workers was 36.5% (95% CI: 31, 42). The absence of immediate treatments for injured health workers (AOR = 8.86, 95% CI: 2.5, 31.4), lack of personal protective equipment (AOR = 3.6, 95% CI: 1.5, 8.4), working greater than eight hours per day (AOR = 7.9, 95% CI: 3.1, 19.7), working in the night shifts (AOR = 8.1, 95% CI: 2.5, 26.1), and absence of effective leadership in the health facility (AOR = 5.2, 95% CI: 1.9, 14.5) were factors associated with the prevalence of occupational hazards.

**Conclusions:**

There was a relatively high degree of occupational health hazard exposure among health workers in the study area compared to kinds of literature from other settings. Health workers were exposed to a wide range of occupational hazards, and risk reduction mechanisms and safety actions were inadequately implemented. Therefore, the health workers' occupational health and safety needs should be prioritized and appropriate measures should be taken to mitigate the problems.

## 1. Background

Worldwide there are approximately sixty million health workers. About two-thirds of them work in healthcare; and the remaining one-third work in management and support. Without them, disease prevention and treatment, as well as advances in healthcare, will be unable to reach, those in need [1]. These health professionals are exposed to various occupational hazards in healthcare institutions; some of them are not aware of exposure and are thus vulnerable to occupational injuries and illnesses. In cases when healthcare workers are aware of the potential occupational hazards at their work sites, mostly personal protective equipment's (PPEs) and other safety devices to mitigate occupational injuries are not available [2].

A large proportion of health workers are exposed to biological, psychological, ergonomic, and chemical hazards in low-income and middle-income settings. However, the implementation of risk reduction measures is suboptimal [3]. It is estimated that 5–7% of global fatalities are attributable to work-related illnesses and occupational injuries [4, 5], and there are about 2.3 million occupationally related deaths associated with work each year [6].

The world health organization (WHO) global burden of disease from occupational hazards among health workers revealed that 37% of the hepatitis B among health workers was the result of occupational exposure and less than 10% of HIV among health workers is the result of exposure at work. Needle stick injuries, the cause of 95% of the HIV occupational seroconversions, are preventable with practical, low-cost measures and have the cobenefit of preventing exposure to other blood-borne viruses and bacteria [7]. A national institute for occupational safety and health report indicated that an estimated 600,000 to 800,000 percutaneous injuries occur annually to healthcare workers [8].

Globally, every year one in ten health professionals sustain a sharp material injury. These sharp material injuries to health professionals end up with sixty-six thousand hepatitis B virus (HBV) infections, one thousand human immunodeficiency virus (HIV) infections, and sixteen thousand hepatitis C virus (HCV) infections. Different scholars have identified that the impact of infections caused by these microorganisms on the few existing health professionals is too high. For instance, it is estimated that these infections will result in 736 premature deaths due to HIV, 145 premature deaths due to HCV, and 261 premature deaths due to HBV by 2030 [7].

Among the thirty-five million health professionals that exist globally, each year around three million are exposed to microorganisms originating from the blood through percutaneous routes because of professional-related accidents [9]. In addition, occupational safety and health administration have determined that nearly five and a half million health professionals working in healthcare facilities are highly susceptible to microorganisms originating from blood including hepatitis C virus, human immune virus, hepatitis B virus, and other potentially infectious materials [10]. The international labor organization (ILO) study showed that occupation-related diseases and injury account for economic losses as high as 4% of the global gross domestic product. Each year greater than three hundred fifty thousand casualties and greater than two million occupational-related mortality occur which are attributable to occupational-related hazards [11].

The mortality rate per 100,000 health professionals is twenty-one and the accident rate is sixteen thousand in sub-Saharan Africa. This means that each year fifty-four health care workers die and forty-two million occupation-related accidents occur that cause at least three working days of absence from a job [12]. Ethiopia is one among underdeveloped countries and does not have much data on the overall occupational hazards. A study conducted in 2008 by the federal civil service agency revealed that 8% of females and 14% of males died, 8% of females and 7% of males were discharged from work due to disability, and 27% of women and 6% of men shifted to other jobs because of different workplace accidents [7].

In the health care setting, system-level problems upsurge the risk of exposure to occupational-related hazards in addition to health professional behaviors. For example, inadequate PPEs, high physician-to-client ratios, and unsafe working environments are among system-level barriers that raise the risk of exposure to blood-borne microorganisms and result in avoidable infections [7]. Occupational health and safety (OHS) procedures have been recognized as efficient means of preventing and controlling associated infections, especially in hospital settings. Such measures not only protect health care workers but also improve the working environment [13].

Evidence related to the magnitude and associated factors of occupational hazards in Ethiopia and the study area is scant. Existing literature has shown a high level of workplace injuries, inadequately organized occupational safety and health services, and limited exposure assessment and monitoring practices [14]. The pooled prevalence of occupational injury in Ethiopia was 44.7% [15]; however, this review included studies that considered workplaces other than the health sector. Another cross-sectional study revealed that nearly half of health professionals had a poor practice of occupational health and safety, and factors including availability of soap and bleach, and availability of infection prevention and control program standards and policy were significantly associated with occupational health and safety of health workers [16]. Undoubtedly the prevalence of occupational injuries in the health care industry will be even higher. This is similar to findings from a different country, the prevalence of occupational hazards among healthcare workers is high and the major contributing factors include the inadequate supply of personal protective equipment, lack of training on occupational health-related hazards and protective measures, chemical splash, needle stick injury, injury from a sharp object, blood contact, standing long period of time, ignorance on health and safety measures, visualizing, sitting, sprain, and strain [17].

Understanding the prevalence of occupational hazards and the contributing factors is very crucial to regional health bureaus, hospital administration, nongovernmental organizations, health care workers, and other researchers to avert problems related to occupational hazards in the study area in particular and in Ethiopia healthcare facilities in general. The evidence can also be relevant for policy adjustment and redesigning strategies for occupational health and safety. Therefore, this paper is designed to assess the magnitude of work-related health hazards and related factors among health professionals in public health institutions in one of the developing regions in Ethiopia (Gambella regional state).

## 2. Methods

### 2.1. Study Setting and Period

The study was conducted in three government health facilities in Gambella town from June 1-21, 2021. Gambella was the capital city of Gambella regional state, which was located 760 kilometers from the capital city of Ethiopia (Addis Ababa). There were two public hospitals in the town, namely, Gambella General Hospital and Gambella town primary hospital, and one health center. Overall, the town's public health facilities had 664 health workers (165 nurses, 40 medical doctors, 40 laboratory professionals, 28 midwives, 18 pharmacists, 2 anesthetics, and 245 supportive staff). Ninety-three of the supportive staffs were cleaners according to data taken from the zonal health department [18].

### 2.2. Study Design and Participants

An institution-based cross-sectional study was undertaken. All selected healthcare workers in the public health facilities of the Gambella town administration, who fulfilled the eligibility criteria, were included in the study. Healthcare workers, who were presented at the time of survey and who had worked in the public health facilities for one and more years, were eligible.

A single population proportion formula was used to calculate the sample size considering the following assumptions: confidence level of 95% was taken, margin of error of 5% (*d* = 0.05) was considered, and the magnitude of occupational hazards among health professionals as 60.1% in a study conducted in Eastern Ethiopia [17]. Since the source population is less than 10, 000, a finite population proportion formula was employed and the corrected sample size yielded 236. Finally, nonresponse rate of 10% was added. Then, the final sampled population was determined to be 260. To select the different categories of health professionals stratified sampling technique was used (stratified by profession). Payroll registration was used as a sampling frame to choose the healthcare worker from each stratum by simple random sampling technique.

### 2.3. Measurement

A semi structured questionnaire was developed based on relevant kinds of literature [3, 4, 9, 10, 16], and adapted to the research objectives. The questionnaire was translated to local language (Amharic) with an expert translator and back-translated to English with independent personnel to maintain consistency. Then, the soft copy tool was uploaded to Open Data Kit (ODK) to collect data. The tool was pretested in thirteen health care workers at nearby public health facilities, and necessary corrections were done as appropriate. Cronbach's alpha was calculated to test the internal consistency of items and the tool had good reliability (Cronbach's alpha between the items of tangibles was 0.841 up to 0.881).

A total of four diploma nurses and two supervisors, who were qualified with bachelor's degrees in public health were selected from outside of the research area and involved in the data collection. Training was given to supervisors and data collectors on the approach to the interviews, details of interviewing techniques, data collection tools, and research ethics. The data collection was conducted at the study facilities after consent was taken from the respondents. Data collection procedures have been monitored on daily basis by supervisors, and necessary feedback had been provided to the data collectors. Furthermore, reviews of completed questionnaires were undertaken every night by a data manager at the central office.

### 2.4. Definition of Variables

The dependent variable was the prevalence of occupational health hazards. Independent variables include socio-demographic and economic factors (sex, age, educational status, marital status, and income), personal factors (stress, smoking, and drinking alcohol), knowledge of occupational hazards (occupational hazard categories, prevention measures of occupational hazard, occupational infections, and source of occupational infection), perception of risk of occupational hazard (needles stick injury, blood/body fluid contact, standing or sitting longer time greater than four hours, and pushing or pulling heavy loads), occupational factors (levels of the health care facility, service year, profession or field of study, working a night shift, wash hands after the procedure, and wearing PPE before work), and environmental factors (lack of PPEs, lack of training, lack of water, and lack good leadership in the facility).

#### 2.4.1. Occupational Health Hazards

Refers to an act that endangers the well-being of health workers if they are exposed to their physical body parts in their working environment, which could impose their lives at risk and pose a greater threat to their security and safety in their future life[19].

#### 2.4.2. Healthcare Workers

One, who deliver care and service to the sick directly as doctors and nurses or indirectly as aids helpers, laboratory technicians, pharmacists, medical waste handlers, and management staff.

#### 2.4.3. Prevalence of Occupational Hazard

The health workers experienced at least one type of occupational hazard such as physical, biological, chemicals, ergonomic, and psychosocial hazards in conditions associated with their work in the past twelve months of the study period.

#### 2.4.4. Biological Hazards

In these contexts, biological hazards mean a biological substance that poses a threat to healthcare workers' example, exposure to blood, needle stick injury and body fluid, exposure to respiratory secretion, and skin lesion.

#### 2.4.5. Chemical Hazard

Injury due to chemical substance examples disinfectants and sterilizing agents.

#### 2.4.6. Ergonomic Hazard

In these contexts, ergonomic hazard means to harm or injury due to work position, for example, standing for greater than four hours at work, sitting for greater than four hours without a backrest, and lifting heavy objects greater than 25 kg.

#### 2.4.7. Physical Hazard

Injury or damage on the body of health workers, for example, cut and wound on the body part, burn, and fractures.

#### 2.4.8. Psychological Hazard

In this context, mental hazard due to verbal assault, physical attack, and sexual harassment.

#### 2.4.9. Knowledge

Awareness about the occupational hazard. The health workers' knowledge was measured by using nine items with a “yes” or “no” responses. Health workers, who correctly responded ≥50% of knowledge questions had good comprehensive knowledge, and who responded <50% of knowledge questions had poor knowledge of occupational hazards [20].

### 2.5. Data Analysis

After checking and correcting errors, the collected data were transferred to SPSS version 25 statistical packages for analysis. Descriptive statistics were used to analyze the characteristics of health workers. Mean and standard deviation were computed for continuous variables and frequency distributions for categorical variables. Crosstab was used to show the relative frequency of socio-demographic and personal characteristics toward the occupational hazard.

Binary logistic regression analysis was undertaken to select variables that may have a high probability to predict outcome variables in further analysis. Those variables with a *p*-value <0.25 were reserved for multivariable analysis. Multivariable logistic regression analysis was used to identify factors associated with the main outcome variable. Variables having a *p*-value ≤0.05 in the multivariable regression analysis were considered as associated factors with occupational hazards at 95% CI. The strength of association between the independent and the outcome variable was measured through adjusted odds ratios (AOR). Variance inflation factor was used to check multicollinearity variables and Hosmer‒Lemeshow goodness of fit was used to check model fitness and the *p*-value was found to be 0.302.

### 2.6. Ethical Consideration

Ethical clearance (reference number: IHRPGY/152/21) and a formal letter were taken from Jimma University Ethical Review Board. Then a letter was submitted to respective Gambella general hospital management, Gambella town primary hospitals, and Gambella town health center to gain support for the study. Prior to administering the questionnaires, the aims and objectives of the study were clarified to the participants and personal consent was obtained from the study participant. Confidentiality and anonymity were ensured throughout the execution of the study.

## 3. Results

### 3.1. Characteristics of Study Participants

A total of 260 health workers were involved in this study with a response rate of 100%. Greater than six in ten of the respondents were from Gambella general hospital 166 (64%) and nearly half 128 (49%) of them were clinical staff. The age range of participants ranged from 22 to 46 with a majority of participants being in the age group of 26–32 (67%). The mean age was 30.7 (SD ± 4.6) and males account for half of 131 (50.4%) health workers. The majority of the health workers 182 (70%) were married and 150 (58%) were protestant religious followers. Regarding their education 214 (82%) have attended higher education and 36 (14%) have attended primary education. Among the health workers, 146 (56%) of them had an average monthly income of greater than 5,500 Ethiopian Birr. Moreover, greater than half or 133 (52%) of the respondents worked more than five years and the average service year of health workers was 5 (SD ± 2.9) (Table 1).

### 3.2. Prevalence of Occupational Hazard

Greater than one-third (36.5%, 95% CI: 30.9–42.5) of the health workers encountered at least one occupational hazard from the five components of hazards (biological, chemical, physical, ergonomic, and psychosocial hazards) in the last one year prior to survey date. Of the overall hazard, psychosocial hazard accounted for half (51.5%) followed by biological hazard (41%), ergonomic hazard (23%), chemical hazard (20%), and physical hazard (12.6%) (Table 2).

### 3.3. Factors Associated with Occupational Hazards

Binary logistic regression analysis was undertaken to select a candidate variable at a *p*-value of <0.25. Of the independent variables identified as a candidate, five variables have shown a statistically significant association with the occupational hazard status of health care workers at the *p*-value <0.05 after adjusting for other variables.

This study found that the odds of occupational hazards were nearly nine times (AOR = 8.86, 95% CI: 2.5–31.4) more likely among health workers, who reported that there were no measures in place to ensure immediate treatments for injured workers compared to those reported as measures were available. In addition, the odds of occupational hazards were four times (AOR = 3.6, 95% CI: 1.5–8.4) more likely among health workers who reported that there was a lack of PPEs in the facility as compared to reported no lack of PPEs in the facility. In terms of working hours, the odds of occupational hazard were nearly eight times (AOR = 7.9, 95% CI: 3.1–19.7) more likely among health workers, who reported working more than eight hours as compared to working less than or equal to eight hours. In the case of working a night shift, the odds of occupational hazard were eight times (AOR = 8.1, 95% CI: 2.5–26.1) more likely among health workers, who reported working a night shift as compared to working daytime. In relation to leadership, the odds of occupational hazard were five times (AOR = 5.2, 95% CI: 1.9–14.5) more likely among health workers, who reported there was no good leadership in the facility as compared to reported there was good leadership (Table 3).

## 4. Discussion

Healthcare facilities like other high-risk workplaces are characterized by a high level of exposure to hazardous agents, which significantly endangers the health and life of health workers. Unsafe conditions in a working environment for health professionals and a high physician-to-client ratio upsurge the risk of exposure to blood-borne microorganisms and resulted in avoidable infections. This study revealed that greater than one-third (36.5%) of the health workers encountered at least one type of occupational hazard in the last 12 months prior to the survey date. This finding was lower than the study done in public health institutions of South India (62%) [21], Jegol hospital in Eastern Ethiopia (60%) [17], and a study done in Kampala, which accounts for 50% [22]. The variations in prevalence of work-related hazards might be because of the difference in the capacity and type of the health institutions, and the composition of health workers considered. In the study area, health center and primary hospital were included, unlike in other settings. In addition, the study period and study participants might contribute to the difference in the magnitude of occupational hazards. In the current study, half of the respondents were management and supportive staff, and as compared to the clinical staff, their probability of getting hazards might be minimized. On the contrary, the prevalence of work-related hazards in the study area was higher than a finding from Wolaita Sodo (19%) [23] by nearly two folds. The variations in the prevalence, in this case, might be because of the difference in work experience of health workers where in the study area almost half of the health workers had work experience of less than five years so the hazard might be increased. In spite of the variations of the magnitude of occupational hazards, the current study finding implies that significant proportion of health workers was at risk of biological, chemical, physical, ergonomic, and psychosocial hazards in the workplaces that require urgent measure to mitigate the problem.

The psychological hazards (51.5%) and biological hazards (41%) were the major occupational hazards among health workers in the study area. This finding was comparable to the findings reported by a study done in north-central Nigeria [24] and Kampala in Uganda [22]. In the current study, the psychological hazards accounted for 18% of the total respondents; and that of a study done in Nigeria accounted 16% [25], and a finding from Kampala in Uganda 22% [22]. On the contrary, the current finding was lower than another study finding from Nigeria (83%) [26], a finding in Jugol Hospital in Eastern Ethiopia (51%) [17] and Northwest Ethiopia (30%) [27]. In the current research 15% of the total health workers were exposed to biological hazards; a finding lower than a study done in Southern India (81%) [21], Uganda (39.5%) [22], Eastern Ethiopia (52.7%) [17], Hawassa city in Southern Ethiopia (35.8%) [28] and Tigray in Northern Ethiopia (25%) [24]. The variations in the magnitude of psychosocial and biological hazards among the health workers might be because of the difference in the health system characteristics, and the type of health workers included in the studies. Health workers in higher setup or specialized hospitals relatively had greater exposure than those in the lower setup like primary hospitals and health centers. Moreover, the clinical staffs were more likely to get biological hazards than nonclinical staff [29, 30].

The current research revealed that the lack of PPEs, absence of measures to ensure immediate treatments to injured workers, working more than eight hours in a day, working in a night shift, and absence of good leadership in the health facility were associated with increased odds of work-related occupational hazards. The healthcare workers who lacked PPEs in the health facility were about four times more likely to get occupational hazards as compared to those who had access to PPEs. This was consistent with study findings from Wolaita in Southern Ethiopia [23] and the University of Gondar Hospital in Northwest Ethiopia [29]. Findings from Uganda and other countries in Africa showed that using PPEs was associated with reduced occupational hazards and PPEs had been long recognized as an important infection control measure in the healthcare industry [22, 31]. This finding suggests that availing of adequate PPEs all time in the health facilities has paramount importance in the reduction of occupational health hazards among health workers.

The health workers, who worked more than eight hours, were about eight times more likely to acquire occupational hazards as compared to those, who were working less than or equal to eight hours. This finding was supported by a study done in low-and-middle-income countries [3] and a study done in central Tigray in Northern Ethiopia [24]. A finding from Tigray reported that health workers, who work greater than 40 hours per week, were sixteen times more likely to experience needle sticks and sharp injury than those, who were working less than or equal to 40 hours per week [24]. Similarly, a study done in black lion hospital in Addis Ababa reported that the health workers, who worked more than 40 hours per week, were two times more likely exposed than those, who were working less than 40 hours per week [22]. Another finding from Uganda revealed that health workers, who worked overtime had increased likelihood of experiencing both biological and nonbiological hazards. Long working hour's results in prolonged exposures to hazards and limited recovery time, which translates into physiologic depletion that continues to the next workday.

Working on the night shift also showed an association with an occupational hazard in those health workers, who worked the night shift, were eight times more likely to get hazards as compared to those, who worked the daytime. This finding was consistent with the study conducted in Northwest Ethiopia, which showed that those, who were working night shift were more likely to be exposed to violence compared to their counterparts [32]. Those working night shifts are more likely to experience workplace violence than their colleagues on day shifts because of low level of security, lower staff, and lower work performance because of feeling insecurity so the patient or attendants were unsatisfied. These initiated conditions are favorable for violence.

The absence of good leadership was also significantly associated with occupational hazards. The health workers, who reported as there was no good leadership in the facility, were five times more likely to be exposed to occupational hazards than those, who reported the presence of good leadership. A similar finding was reported by a study done in Hawassa city in Sothern Ethiopia, which showed that poor leadership was associated with higher exposure of health workers to needle stick injury in the facility [28]. These could be due to the fact that in health facilities with poor leadership the leader might not supply a sufficient amount of PPEs, be unable to prepare insight training, and do not implement rules and procedures at the worksite which in turn exposes the workers to an occupational hazard.

The health workers, who had reported the absence of measures in place to ensure immediate treatments for injured workers were about nine times more likely to get hazards as compared to those, who responded as there was a measure in place. Immediate treatment measures and safety for injured health workers can prevent further transmission and exacerbation of occupational hazards, which endangers the life of health professionals as delivery of quality health care depends largely on the quality of staff delivering these services.

### 4.1. Strength and Limitations of the Study

As a strength, the study has considered the different categories of health workers (the clinicians and support staff) to examine the prevalence of work-related health hazards, and the different categories of occupational hazards were assessed. A pretested questionnaire was used and data collection was assisted by the Open Data Kit (ODK), which increases the quality of data. As a limitation, this study employed a cross-sectional study design that capture a snapshot of a certain event at a certain point in time. So, causal relationships between dependent and independent variables were not assumed. The previous exposure status of health workers was assessed and thus this might lead to a recall bias.

## 5. Conclusions

This study concluded that there was a high degree of occupational hazard exposure among the health workers in the study area compared to kinds of literature in other parts of the World and in Ethiopia. Poor leadership in the healthcare facilities, lack of PPEs, longer working hours per day, working on a night shift, and the lack of immediate treatments for injured health workers were the predictors of occupational hazards in the study area. The health workers in the study area were exposed to a wide range of occupational hazards and the risk reduction mechanisms and safety actions were inadequately implemented mainly due to the lack of PPEs, poor leadership and workers staying in worksites for a longer period of time and overnight. To protect health care workers in this study area and elsewhere in the country, first and foremost, occupational health and safety need to be prioritized. Therefore, we strongly recommend that policymakers, health leaders, health Managers, regional health bureaus, healthcare planners, and zonal health departments should devise measures to improve health care employees' working conditions and expand their access to personal protective equipment in order to protect them from occupational injuries.

## Figures and Tables

**Table 1:** Characteristics of healthcare workers in health facilities of Gambella town, Western Ethiopia, 2021 (*N* = 260).

Variables	Category	Frequency (%)	Hazard status	
			Yes (*n*, (%))	No (*n*, (%))
Facility type	Gambella general hospital	166 (63.8)	41 (43.2)	125 (75.8)
	Gambella town primary hospital	74 (28.5)	41 (43.2)	33 (20)
	Gambella town health center	20 (7.7)	13 (13.6)	7 (4.2)

Sex	Male	131 (50.4)	51 (53.7)	80 (48.5)
	Female	129 (49.6)	44 (46.3)	85 (51.5)

Age	<30	122 (46.9)	49 (51.6)	73 (44.2)
	≥30	138 (53.1)	46 (49.4)	92 (55.8)

Marital status	Single	70 (26.9)	34 (35.8)	36 (21.6)
	Married	182 (70)	58 (61.1)	124 (75.3)
	Divorced	8 (3.1)	3 (3.1)	5 (3.1)

Religion	Orthodox	78 (30)	30 (31.6)	48 (29.1)
	Muslim	32 (12.3)	16 (16.8)	16 (9.7)
	Protestant	150 (57.7)	49 (51.6)	101 (61.2)

Profession	Medical doctors	22 (8.5)	7 (7.4)	15 (9.1)
	Management staff	86 (33.1)	14 (14.7)	72 (43.6)
	Nurse	64 (24.6)	38 (40)	26 (15.8)
	Cleaner	46 (17.7)	14 (14.7)	32 (19.4)
	Others	42 (16.2)	22 (23.2)	20 (12.1

Average monthly income	≤5500 birr	114 (43.8)	40 (42.1)	74 (44.8)
	>5500 birr	146 (56.2)	55 (57.9)	91 (55.2)

Service experience in years	≤5 years	127 (48.2)	54 (56.8)	73 (44.2)
	>5 years	133 (51.8)	41 (43.2)	92 (55.8)

**Table 2:** Prevalence of occupational hazards among health workers.

Variables	Frequency (%)
Prevalence of work hazard	95 (36.5)
Ever had an incident of biological hazard in the job in the last 12 months	39 (15)

Type of biological hazard faced by the health workers	
Needle stick injury	11 (28.2)
Blood exposure	11 (28.2)
Body fluid exposure	7 (17.9)
Respiratory secretion	7 (17.9)
Infected skin lesion contact	3 (7.7)

Causes of injury	
Patient movement during injection	4 (10.3)
During recapping	9 (23.1)
Lack of use of PPEs	15 (38.5)
Due to the carelessness of healthcare workers	5 (12.8)
Others	6 (15.4)
Ever had a chemical hazard incident in the job in the last 12 months	19 (7.3)

Types of chemical hazards encountered by the health workers	
Disinfectant	8 (42.1)
Contact a sterilizing agent	9 (47.4)
Others	2 (10.5)

Causes of chemical hazard	
Due to the carelessness of HCWs	2 (10.5)
During cleaning	13 (68.4)
Lack of use of PPEs	4 (21)
Ever had a physical hazard incident at a job in the last 12 months	12 (4.6)

Types of physical hazards encountered by the health workers	
Sharp material related injury	7 (58.3)
Cut and wound	4 (33.3)
Burn	1 (8.3)

Causes of physical hazard	
Unintended movement of the patient during care	7 (58.4)
Lack of use of PPEs	1 (8.3)
Due to the carelessness of HCWs	1 (8.3)
The difficulty of an object to use	3 (25)
Ever had an ergonomic hazard incident in the job in the last 12 months	22 (8.5)

Types of ergonomic hazards encountered by HCWs	
Back pain	19 (86.4)
Strain or sprain	3 (13.6)

Causes of ergonomic hazard	
Due to long-standing	16 (72.7)
Sprain and strain	1 (4.5)
Due to sitting without a back seat	5 (22.7)
Lifting a heavy object or patient greater than 25 kg	146 (56.2)
Standing greater than 4 hours at work	153 (58.8)
Ever had a psychosocial hazard incident in the job in the last 12 months	49 (18.8)

Types of psychological hazards encountered by the HCWs	
Verbal abuse	43 (87.8)
Physical attack	5 (10.2)
Sexual harassment	1 (2)

Physiological challenges currently being experienced by the healthworkers that are resulting from work-related hazards	
Loss of sleep due to stress from work	17 (34.7)
Persistent tiredness due to work activities	27 (55.1)
Fatigue	2 (4.1)
Social relationships due to many hours spent at work	3 (6.1)

**Table 3:** Factors associated with occupational hazards.

Variable	Occupational hazard		COR (95% CI)	AOR (95% CI)
	Yes	No		
Level of health care facility				
Gambella GH	41	125	1	1
Gambella town PH	41	33	0.18 (0.1–0.5)	0.28 (0.48–1.65)
Gambella town HC	13	7	0.67 (0.2–1.9)	1.28 (0.23–7.3)

Time in hours that passed on work/day				
Less than or equal to 8 hours	27	107	1	1
Greater than 8 hours/day	68	58	4.65 (2.7–8.0)	**7.9** (**3.1**–**19.7**)^*∗∗*^
Working night shift				
Yes	74	77	4.03 (2.3–7.1)	**8.1** (**2.5**–**26.1**)^*∗∗*^
No	21	88	1	1

Do you have conducive working environments				
Yes	42	99	1	1
No	53	66	1.89 (1.1–3.2)	0.31 (0.08–1.19)

Are there measures in place to ensure immediate treatment for injured health workers?				
Yes	30	101	1	1
No	65	64	3.42 (2.0–5.8)	**8.9** (**2.5**–**31.4**)^*∗∗*^

Lack of personal protective equipment in the facility?				
Yes	50	56	2.16 (1.3–3.6)	**3.6** (**1.5**–**8.4**)^*∗*^
No	45	109	1	1

Lack of water in the facility?				
Yes	53	139	0.24 (0.1–0.4)	0.22 (0.07–0.68)
No	42	26	1	1

Is there effective leadership in the facility?				
Yes	43	118	1	1
No	52	47	3.04 (1.8–5.1)	**5.21** (**1.9**–**14.4**)^*∗*^

Is there a lack of lifting transportation of patients in the facility?				
Yes	25	103	1	1
No	70	62	4.62 (2.7–8.1)	0.51 (0.12–2.14)

Lack of information regarding the use of modern tools and equipment in the facility?				
Yes	24	98	1	1
No	71	67	4.33 (2.5–7.6)	2.56 (0.25–9.60)

Is there a lack of policies and procedures for occupational safety in the facility?				
Yes	19	109	1	1
No	76	56	7.79 (4.3–14.1)	0.78 (0.16–3.74)

Do the waste management workers get safety training?				
Yes	60	129	1	1
No	35	36	2.09 (1.2–3.6)	0.96 (0.26–3.51)

Do regular supervision practices exist by management team in health facilities				
Yes	42	112	1	1
No	53	53	0.38 (0.2–0.6)	0.97 (0.29–3.23)

Respect to rest breaks hours observed in the workplace				
Yes	80	158	1	1
No	15	7	4.23 (1.7–10.8)	2.43 (0.75–5.56)

Training on occupational health and safety				
Yes	34	96	1	1
No	61	69	2.45 (1.5–4.2)	0.56 (0.35–4.2)

Perception of risk of occupational hazard				
Good	45	45	1	1
Poor	50	120	2.40 (1.4–4.1)	1.41 (0.46–4.36)

Knowledge of respondents				
Good	36	114	1	1
Poor	59	51	3.66 (2.2–6.2)	1.46 (0.50–4.28)

Personal safety provision and related factors				
Good	58	122	1	1
Bad	37	43	0.55 (0.3–0.9)	2.98 (0.9–8.91)

*Note.* ^*∗*^ denotes statistical significance at *P* < 0.05 and ^*∗∗*^ denote statistical significance at *P* < 0.01. abbreviations: AOR: adjusted odd ratio; COR: crude odds ratio; CI: confidence interval; GH: general hospital; PH: primary hospital; HC: health center; 1: referred to reference category. The bold values show independent variables that had significant association with dependent variables (Occupational health hazards).

## Data Availability

The datasets used and/or analyzed during the current study are not openly available because data are part of the ongoing research project and available from the corresponding author upon reasonable request.
